The article "Meta-analysis of the Efficacy of the Anatomical Center and High Hip Center Techniques in the Treatment of Adult Developmental Dysplasia of the Hip" was published in 2022. Journal: Biomed Res Int.

# Meta-analysis of the Efficacy of the Anatomical Center and High Hip Center Techniques in the Treatment of Adult Developmental Dysplasia of the Hip

**DOI:** 10.1155/2022/7256664

**Published:** 2022-08-30

**Authors:** Chen Wu, Guoyin Shu, Xiaowei Xie, Xin Yuan, Shirong Chen

**Affiliations:** Department of Orthopaedic Surgery, Second Affiliated Hospital of Chongqing Medical University, Chongqing, China

## Abstract

**Background:**

In total hip arthroplasty for the treatment of adult developmental dysplasia of the hip, there is considerable controversy regarding the placement of the acetabular cup, anatomic center, and upward in acetabular reconstruction. This article explores the efficacy of the anatomical center technique and high hip center technique in the treatment of adult developmental dysplasia of the hip.

**Method:**

By searching for articles in the Cochrane Library, PubMed, CNKI, and Wanfang databases, we collected the literature on the treatment of adult developmental dysplasia of the hip by anatomical center and high hip center technology and screened the literature according to the inclusion and exclusion criteria. The Cochrane risk of bias assessment tool was used to assess the risk of bias of randomized controlled trials, the quality of the literature in retrospective cohort studies was assessed using the Newcastle–Ottawa scale, and the RevMan 5.4 software was used to analyze the extracted outcome indicators.

**Results:**

Nine studies were finally included, including one prospective cohort study, eight retrospective cohort studies, two high-quality studies, and six moderate-quality studies. The meta-analysis results showed that the reconstruction of the acetabulum in two positions was significantly different in terms of operation time (WMD = −37, 95% CI: -45.25-28.74, *P* < 0.00001), intraoperative blood loss (WMD = −91.88, 95% CI: -108.57-75.19, *P* < 0.00001), postoperative drainage volume (WMD = 80.55, 95% CI: -140.56-301.66, *P* = 0.48), time to ground (WMD = −0.68, 95% CI: -1.37-0.0, *P* = 0.05), Harris score (WMD = −0.04, 95% CI: -0.91-0.82, *P* = 0.92), lower limb length difference (WMD = 0.21, 95% CI: -0.22-0.64, *P* = 0.33), WOMAC score (WMD = −1.24, 95% CI: -4.89-2.41, *P* = 0.51), postoperative complications (RD = −0.02, 95% CI: -0.06-0.02, *P* = 0.44), Trendelenburg sign (RD = −0.02, 95% CI: -0.02-0.05,*P* = 0.31), limb lengthening (WMD = 0.85, 95% CI: 0.61-1.09, *P* < 0.00001), prosthesis wear (WMD = 0.01, 95% CI: 0-0.02, *P* = 0.17), and prosthesis loosening (RD = 0.01, 95% CI: -0.02-0.04, *P* = 0.45).

**Conclusions:**

The high hip center technique can reduce operative time, intraoperative blood loss, and downtime. The anatomical center technique is superior to the high hip center technique in terms of limb lengthening. Compared with acetabular anatomical reconstruction, there was no significant difference in postoperative drainage, lower limb length difference, postoperative complications, Trendelenburg sign, and prosthesis survival or wear. For DDH patients who are not severely shortened in the lower limbs and have severe acetabular bone defects, joint surgeons can choose to reconstruct the acetabulum in the upper part to simplify the operation, reduce the trauma of the patient, and accelerate the recovery of the patient, and they can choose to adjust the length of the neck and the angle of the neck shaft to maintain the moment arm of the abductor muscle. A ceramic interface or a highly cross-linked polyethylene interface minimizes the effect of hip response forces. To further evaluate the efficacy of the anatomical center technique and the high hip center technique in the treatment of adult developmental dysplasia of the hip, more large-sample, high-quality, long-term follow-up randomized controlled trials are still needed for verification.

The article "Meta-analysis of the Efficacy of the Anatomical Center and High Hip Center Techniques in the Treatment of Adult Developmental Dysplasia of the Hip" was published in 2022. Journal: Biomed Res Int.

## 1. Introduction

Developmental dysplasia of the hip is due to abnormal acetabular development leading to poor acetabular inclusion of the femoral head, and long-term biomechanical changes lead to severe osteoarthritis, accompanied by different degrees of femoral head dislocation and acetabular bone loss. Total hip arthroplasty is one of the most effective ways to manage end-stage pain, improve function, and improve quality of life in patients with hip osteoarthritis. Severe acetabular bone defects pose great challenges to joint surgeons, and there has been controversy over whether the acetabulum should be reconstructed anatomically or high. Some scholars believe that the upward placement of the acetabular cup alters the biomechanics of the hip joint, accelerating prosthesis wear, limb shortening, and abductor failure [1–6]. Others believe that the upper internal cup is placed, and the neck stem angle and neck length can be adjusted within an appropriate range to maintain the abductor muscle arm [6]. With the improvement of the prosthesis technology, it has a great impact on the response force of the joint. The magnitude of reduction [7] and the wear of the prosthesis were not significantly different from those of anatomic center reconstruction [8, 9].

The research subject of this article is adult developmental dysplasia of the hip treated by total hip arthroplasty. The anatomical center technique and the high hip center technique were compared, and a meta-analysis of the outcome indicators after total hip arthroplasty was performed. The efficacy of this surgical technique provides more evidence-based medical evidence for the treatment of adult developmental dysplasia of the hip.

The article "Meta-analysis of the Efficacy of the Anatomical Center and High Hip Center Techniques in the Treatment of Adult Developmental Dysplasia of the Hip" was published in 2022. Journal: Biomed Res Int.

## 2. Materials and Methods

### 2.1. Literature Search Strategy

#### 2.1.1. Searcher

The first author performed the literature search.

#### 2.1.2. Search Databases

Data were obtained from Cochrane Library, MEDLINE, PubMed, CNKI, and Wanfang databases.

#### 2.1.3. Search Terms

The search terms were (Anatomic Hip Center) OR (High Hip Center) AND (Developmental Dysplasia of the Hip OR Hip Dislocation, Developmental OR Developmental Hip Dislocations OR Dislocation, Developmental Hip OR Developmental Hip Dislocation OR Developmental Hip Dysplasia OR Developmental Hip Dysplasias OR Dysplasia, Developmental Hip OR Hip Dysplasia, Developmental) AND (Arthroplasty, Replacement, Hip OR Arthroplasties, Replacement, Hip OR Arthroplasty, Hip Replacement OR Hip Prosthesis Implantation OR Hip Prosthesis Implantations OR Implantation, Hip Prosthesis OR Prosthesis Implantation, Hip OR Hip Replacement Arthroplasty OR (Replacement Arthroplasties, Hip OR Replacement Arthroplasty, Hip OR Arthroplasties, Hip Replacement OR Hip Replacement Arthroplasties OR Hip Replacement, Total OR Total Hip Replacement OR Total Hip Arthroplasty OR Arthroplasty, Total Hip OR Hip Arthroplasty, Total).

#### 2.1.4. Search Time Range

The retrieved articles were not subject to publication time constraints.

#### 2.1.5. Literature Search Strategy

The search was performed using subject headings and free words, taking PubMed as an example (see Table 1 for details).

### 2.2. Inclusion and Exclusion Criteria

#### 2.2.1. Inclusion Criteria

The included literature follows the PICO principles: (1) research subjects: adult developmental dysplasia of the hip with secondary osteoarthritis and total hip replacement for the first time. (2) The high hip center technique was used in the experimental group during total hip arthroplasty, while the anatomical center technique was used in the control group during total hip arthroplasty. (3) Control comparison: the patients treated with the high hip center technique were compared with the patients treated with the anatomical center technique. (4) Outcome indicators: the main outcome indicators were operation time, intraoperative blood loss, postoperative drainage volume, postoperative complications, time to the ground, lower limb length difference, limb lengthening, Harris score, WOMAC score, Trendelenburg sign, prosthesis wear rate, and prosthesis loosening rate. (5) Type of literature: the meta-analysis included randomized controlled trials, case–control studies, and cohort studies using anatomical center techniques and high hip center techniques in adults with developmental dysplasia of the hip secondary to osteoarthritis for the first time in total hip replacement.

The article "Meta-analysis of the Efficacy of the Anatomical Center and High Hip Center Techniques in the Treatment of Adult Developmental Dysplasia of the Hip" was published in 2022. Journal: Biomed Res Int.

#### 2.2.2. Exclusion Criteria

The exclusion criteria are as follows: (1) studies without a control group; (2) studies with a severe lack of literature data; and (3) case reports, conference papers, reviews, and other literature.

### 2.3. Data Extraction and Processing

Relevant documents retrieved from the databases were imported into NoteExpress 3.4, and duplicate documents were removed through the software's functions. Two professionally trained researchers read the titles and abstracts of the literature for preliminary screening, and the remaining studies were read in full text and further screened according to the inclusion and exclusion criteria. A table for extracting data and information was made. Disputes were resolved through discussion with a third senior orthopedic physician.

### 2.4. Literature Quality Evaluation

This study followed the requirements of the PRISMA (Preferred Reporting Items for Systematic Reviews and Meta-Analyses) statement [10]. The risk of bias for randomized controlled trials was assessed using the Cochrane Risk of Bias Tool (https://www.cochraneIibrary.com/). The quality of the retrospective cohort studies was evaluated using the Newcastle–Ottawa scale. The full score of this scale is 9 points, ≥7 indicates high-quality literature, 5-6 indicates medium-quality literature, and <5 indicates low-quality literature. The first author of this article and a senior orthopedic physician independently evaluated the quality of the literature. If there was a disagreement, the third orthopedic chief physician evaluated the quality of the literature.

### 2.5. Outcome Indicators

(1) General information of the literature is as follows: first author, country, publication year, research type, sample size, average age, follow-up period, and so on. (2) Outcome indicators are as follows: operation time, intraoperative blood loss, postoperative drainage volume, postoperative complications, time to descend, lower limb length difference, limb lengthened length, Harris score, WOMAC score, Trendelenburg sign, prosthesis wear, prosthesis loosening, horizontal distance from the center of rotation to the teardrop, vertical distance from the center of rotation to the teardrop, and cost of hospitalization.

### 2.6. Statistical Analysis

The meta-analysis was performed using RevMan 5.4. In this paper, the number of occurrences in the experimental group and the control group was 0 in the binary variables of some literature in this paper, which cannot be expressed by the odds ratio (OR) or the relative risk expression (RR); thus, the risk difference (RD) and 95% confidence interval (CI) were used, such as for postoperative complications, the Trendelenburg sign, and prosthesis loosening. Continuous variables, such as operation time, intraoperative blood loss, postoperative drainage, lower limb length difference, limb lengthening, Harris score, WOMAC score, and prosthesis wear, were expressed by the mean difference (WMD) or standardized mean (SMD) expression and 95% confidence interval (CI). When *P* ≥ 0.1 or *I*^2^ ≤ 50, the homogeneity was considered to be good, and the fixed-effects model was used for analysis; when *P* < 0.1 or *I*^2^ > 50, the heterogeneity was considered to be large, the random-effects model was used for analysis, and a subgroup analysis or sensitivity analyses identified sources of heterogeneity.

The article "Meta-analysis of the Efficacy of the Anatomical Center and High Hip Center Techniques in the Treatment of Adult Developmental Dysplasia of the Hip" was published in 2022. Journal: Biomed Res Int.

## 3. Results

### 3.1. Literature Search Results and Process

A total of 845 related studies were retrieved from five Chinese and foreign databases (Cochrane Library, MEDLINE, PubMed, CNKI, and the Wanfang databases), and 9 studies were finally included. The detailed screening process is shown in Figure 1. The basic characteristics of the included studies are shown in Table 2.

### 3.2. Quality Assessment and Risk of Bias of Included Studies

Nine studies with a total of 571 patients were included, including 288 patients using the high hip center technique and 283 patients using the anatomical center technique. One randomized controlled trial assessed the quality of the literature according to the risk of bias assessment criteria recommended by the Cochrane Handbook (Figures 2 and 3). Eight retrospective cohort studies were assessed by the NOS scale, of which 2 were of high quality and 6 were of moderate quality (see Table 3).

### 3.3. Meta-Analysis Results

#### 3.3.1. Differences in Operation Time between Groups

Three included studies compared operative time [14–16]. The meta-analysis results showed significant heterogeneity (*I*^2^ = 85%, *P* = 0.001). A sensitivity analysis was performed to find the source of heterogeneity. After excluding the literature by Zhang et al. [14], the heterogeneity decreased most significantly (*I*^2^ = 66%). However, there was still significant heterogeneity. From a careful reading of the full text, it may be related to the fewer cases of structural bone grafting in the control group, but Zhang et al. [14] separately analyzed the placement of structural bone grafts. The high hip center technique significantly increased the operation time (average 250 minutes vs. 145 minutes) [14]. Therefore, the random-effects model analysis was used, and the results showed that the operation time of the high hip center technique and the anatomical center technique was shorter (WMD = −37, 95% CI: -45.25-28.74, *P* < 0.00001), as shown in Figure 4.

The article "Meta-analysis of the Efficacy of the Anatomical Center and High Hip Center Techniques in the Treatment of Adult Developmental Dysplasia of the Hip" was published in 2022. Journal: Biomed Res Int.

#### 3.3.2. Differences in Intraoperative Blood Loss between the Groups

Three included studies compared intraoperative blood loss [14–16]. The meta-analysis showed slight heterogeneity (*I*^2^ = 31%, *P* = 0.23) using a fixed-effects model. The results showed that compared with the anatomical center technique, the high hip center technique had less intraoperative blood loss (WMD = −91.88, 95% CI: -108.57-75.19, *P* < 0.00001), as shown in Figure 5.

#### 3.3.3. Differences in Postoperative Drainage Volume between Groups

Two included studies compared the postoperative drainage volume [14, 16]. The meta-analysis results showed significant heterogeneity (*I*^2^ = 83%, *P* = 0.02), so a random-effects model was used. The results showed no significant difference in postoperative drainage between the high hip center technique and the anatomical center technique (WMD = 80.55, 95% CI: -140.56-301.66, *P* < 0.48) (see Figure 6).

#### 3.3.4. Differences in the Time of Going to the Ground between Groups

In the included studies, two studies compared the time of going to the ground [14, 16]. The meta-analysis results showed no significant heterogeneity (*I*^2^ = 0%, *P* = 0.67) using a fixed-effects model. The results showed that the time spent on the ground in patients with the high hip center technique was less than that in the anatomical center technique (WMD = −0.68, 95% CI: -1.37-0.0, *P* = 0.05) (see Figure 7).

#### 3.3.5. Differences in Postoperative Harris Scores between Groups

Seven included studies compared postoperative Harris scores [8, 12–17]. The meta-analysis results showed slight heterogeneity (*I*^2^ = 24%, *P* = 0.24) using a fixed-effects model. The results showed no significant difference in the postoperative Harris score between the high hip center technique and the anatomical center technique (WMD = −0.04, 95% CI: -0.91-0.82, *P* = 0.92) (see Figure 8).

#### 3.3.6. Differences in Limb Length Difference between the Groups

Five of the included studies compared differences in limb length difference [12, 14–17]. The meta-analysis showed no significant heterogeneity (*I*^2^ = 0%, *P* = 0.63) using a fixed-effects model. The results showed no significant difference in limb length between the high hip center technique and the anatomical center technique (WMD = 0.21, 95% CI: -0.22-0.64, *P* = 0.33) (see Figure 9).

#### 3.3.7. Differences in WOMAC Scores in Each Group

Two of the included studies compared postoperative WOMAC scores [11, 14]. The meta-analysis results showed no significant heterogeneity (*I*^2^ = 0%, *P* = 0.53) using a fixed-effects model. The results showed no significant difference in the postoperative WOMAC score between the high hip center technique and the anatomical center technique (WMD = −1.24, 95% CI: -4.89-2.41, *P* = 0.51) (see Figure 10).

The article "Meta-analysis of the Efficacy of the Anatomical Center and High Hip Center Techniques in the Treatment of Adult Developmental Dysplasia of the Hip" was published in 2022. Journal: Biomed Res Int.

#### 3.3.8. Differences in Postoperative Complications between Groups

Seven included studies compared postoperative complications [8, 11–14, 16, 17]. The meta-analysis results showed no significant heterogeneity (*I*^2^ = 0%, *P* = 0.94) using a fixed-effects model. The results showed no significant difference between the high hip center technique and the anatomical center technique in terms of postoperative complications (RD = −0.02, 95% CI: -0.06-0.02, *P* = 0.44) (see Figure 11).

#### 3.3.9. Differences in the Postoperative Trendelenburg Sign between Groups

Six included studies compared the postoperative Trendelenburg sign [8, 12, 13, 15–17]. The meta-analysis results showed no significant heterogeneity (*I*^2^ = 0%, *P* = 0.81) using a fixed-effects model. The results showed no significant difference between the high hip center technique and the anatomical center technique in terms of the postoperative Trendelenburg sign (RD = −0.02, 95% CI: -0.02-0.05, *P* = 0.31) (see Figure 12).

#### 3.3.10. Differences in the Length of Limb Lengthening between Groups

Two of the included studies compared limb lengthening [8, 14]. The meta-analysis showed heterogeneity (*I*^2^ = 49%, *P* = 0.16) using a fixed-effects model. The results showed that the anatomical center technique was superior to the high hip center technique in terms of limb lengthening (WMD = 0.85, 95% CI: 0.61-1.09, *P* < 0.00001), as shown in Figure 13.

#### 3.3.11. Differences in Prosthesis Wear in Each Group

Two of the included studies compared prosthesis wear [8, 9]. Meta-analysis results showed no significant heterogeneity (*I*^2^ = 0%, *P* = 0.6) using a fixed-effects model. The results showed no significant difference in prosthesis wear between the high hip center technique and the anatomical center technique (WMD = 0.01, 95% CI: 0-0.02, *P* = 0.17) (see Figure 14).

#### 3.3.12. Differences in Prosthesis Loosening in Each Group

Five of the included studies compared prosthesis wear [11, 13, 15–17]. The meta-analysis showed no significant heterogeneity (*I*^2^ = 0%, *P* = 0.85) using a fixed-effects model. The results showed no significant difference in prosthesis loosening between the high hip center technique and the anatomical center technique (RD = 0.01, 95% CI: -0.02-0.04, *P* = 0.45) (see Figure 15).

## 4. Discussion

### 4.1. Summary of the Evidence

Adult DHH is prone to secondary osteoarthritis, which significantly reduces the quality of life of patients. At present, total hip replacement is one of the most important treatment methods. The purpose of its treatment is to improve the function of the hip joint and relieve pain. However, acetabular reconstruction is still an important challenge for patients with Crowe II and III DHH. Anatomical reconstruction of the acetabulum can reduce the stress of the hip joint, avoid the failure of the abductor muscles, and effectively restore the length of the lower extremity. Anatomical reconstruction of the acetabulum can reduce the stress of the hip joint, avoid the failure of the abductor muscles, and effectively restore the length of the lower limb, but the disadvantage is that structural bone grafting is needed, which greatly increases the difficulty of the operation, the operation time, and the trauma to the patient. High hip center technology can achieve effective bone coverage of the acetabular cup, avoid structural bone grafting and the possibility of related complications such as bone resorption and bone nonunion after bone grafting, simplify the operation difficulty, and reduce the operation time, intraoperative blood loss, and surgery costs. However, it changes the biomechanics of the hip joint. Therefore, whether to choose anatomical reconstruction or high placement for the treatment of adult DHH has always been an issue for joint surgeons to consider.

The article "Meta-analysis of the Efficacy of the Anatomical Center and High Hip Center Techniques in the Treatment of Adult Developmental Dysplasia of the Hip" was published in 2022. Journal: Biomed Res Int.

This study included one randomized controlled study and eight retrospective, controlled studies for a meta-analysis. Studies have shown that the anatomical center technique has a longer operative time and more intraoperative blood loss. The reason is that to increase the cup coverage, structural bone grafting or the use of tantalum trabecular bone reinforcement technology is needed, thus increasing the difficulty and time of the operation. The results of the operation time analysis showed obvious heterogeneity. The sensitivity analysis of the literature and the exclusion of the literature by Zhang et al. [14] could reduce the heterogeneity, but there was still significant heterogeneity, which may be inconsistent with the surgeon's proficiency in surgery. The proficiency of surgical assistants and instrument nurses was inconsistent, and the standard of operation time recording was different. Although only two studies mentioned the postoperative drainage volume, the results of the analysis showed no significant difference between the experimental group and the control group, and there was obvious heterogeneity. The reasons may be related to the use of hemostatic drugs and the dose of anticoagulant drugs during the perioperative period, intraoperative soft tissue release and clearance of surrounding osteophytes, and the coagulation function of patients. The cost of hospitalization was only mentioned in the literature by Zhang et al. [14]. The argument is weak and not used as the primary outcome measure, but the results show that the high hip center technique costs an average of $270 less than the anatomical center technique [14].

The article "Meta-analysis of the Efficacy of the Anatomical Center and High Hip Center Techniques in the Treatment of Adult Developmental Dysplasia of the Hip" was published in 2022. Journal: Biomed Res Int.

The meta-analysis forest plot showed no significant differences in the lower extremity length difference, postoperative complications, prosthesis wear, prosthesis loosening, WOMAC score, Harris score, or Trendelenburg sign. Stirling et al. [18] systematically reviewed 475 cases of total hip arthroplasty due to osteoarthritis secondary to DDH (207 cases with cup upward placement and 268 cases with cup anatomical reconstruction). The results showed no significant differences in Harris scores and revision rates. These findings are consistent with the conclusions of this study. However, some studies contradict the results of this paper. Karaismailoglu et al. [19] and other studies believe that high hip center technology will increase the load of the hip joint and reduce the dynamic range of motion, thereby reducing the survival rate of the prosthesis and increasing the risk of falls. Research by Fukushi et al. [20] showed that the high hip center technique significantly delayed the recovery of abductor muscle strength. Due to the short follow-up time of the included articles, more high-quality, long-term follow-up studies need to be included for analysis.

At present, there is no uniform standard for the upward placement of the acetabular cup in the high hip center technique. Russotti and Harris [21] first proposed the use of a high hip center technique in hip revision surgery and defined the standard as 35 mm from the teardrop from the center of rotation. The study by Kaneuji et al. [22] used an acetabular cup distance of 20 mm from the teardrop as the standard for the high hip center of Crowe I-III-type DDH. Schutzer and Harris [23] set the standard as 25 mm. In many studies, the standard of a high hip center for the first total hip arthroplasty in DDH is that the acetabular cup is more than 30 mm from the teardrop [8, 24–26], and this standard is also widely recognized and used in surgery by joint surgeons. However, there was obvious heterogeneity in the vertical distance and horizontal distance of the postoperative rotation center in this paper, and the subgroup analysis and sensitivity analysis could still could not eliminate or significantly reduce the heterogeneity. This may be related to the selection of different high hip center technology placement standards, different reference anatomical landmarks, or differences in pelvic anatomy between different races, which may have a certain impact on the center of rotation and whether it is placed inward. Therefore, it was not used as the primary outcome indicator. More high-quality research needs to be included in the future to further improve the high-level placement standard between different races.

The article "Meta-analysis of the Efficacy of the Anatomical Center and High Hip Center Techniques in the Treatment of Adult Developmental Dysplasia of the Hip" was published in 2022. Journal: Biomed Res Int.

### 4.2. Limitations of the Paper

There are certain limitations of this study: (1) this study only searched five commonly used Chinese and English databases, and the literature search may not have been sufficiently comprehensive. (2) When extracting data, some studies were excluded due to language, lack of data, and other reasons, leading to the defect of fewer included studies. (3) The quality of the evidence was rated high in only two studies. This reduces confidence in the findings. However, this might be more of a concern if the results of the review were more positive as it could be argued that lower quality evidence may be more subject to bias. (4) The follow-up time of some cases in the literature was short and inadequate for judging the long-term efficacy. (5) Most of the patients included in this study were Crowe I-III patients who had received interventions for high hip or anatomical center reconstruction of the acetabulum, so the results of this study can only be generalized to Crowe I-III patients.

## 5. Conclusions

The high hip center technique can reduce operative time, intraoperative blood loss, and downtime. The anatomical center technique is superior to the high hip center technique in terms of limb lengthening. Compared with acetabular anatomical reconstruction, there was no significant difference in postoperative drainage, lower limb length difference, postoperative complications, Trendelenburg sign, and prosthesis survival or wear. When treating DDH patients who are not severely shortened in the lower limbs and who have severe acetabular bone defects, joint surgeons can choose to reconstruct the acetabulum in the upper part to simplify the operation, reduce the trauma of the patient, and accelerate the recovery of the patient, and they can choose to adjust the length of the neck and the angle of the neck shaft to maintain the moment arm of the abductor muscle. A ceramic interface or a highly cross-linked polyethylene interface minimizes the effect of hip response forces. To further evaluate the efficacy of the anatomical center technique and the high hip center technique in the treatment of adult developmental dysplasia of the hip, more large-sample, high-quality, long-term follow-up randomized controlled trials are still needed for verification.

The article "Meta-analysis of the Efficacy of the Anatomical Center and High Hip Center Techniques in the Treatment of Adult Developmental Dysplasia of the Hip" was published in 2022. Journal: Biomed Res Int.

## Figures and Tables

**Figure 1:** Article screening process.

**Figure 2:** Risk of bias in randomized controlled trials.

**Figure 3:** Summary of bias in randomized controlled trials.

**Figure 4:** Meta-analysis forest plot for comparison of operation time between two groups.

**Figure 5:** Meta-analysis forest plot for the comparison of intraoperative blood loss between the two groups.

**Figure 6:** Meta-analysis forest plot for comparison of postoperative drainage between the two groups.

**Figure 7:** Meta-analysis forest plot for the comparison of the two groups of the time of going to the ground.

**Figure 8:** Meta-analysis forest plot for comparison of postoperative Harris scores between the two groups.

**Figure 9:** Meta-analysis forest plot for comparison of limb length difference between the two groups.

**Figure 10:** Meta-analysis forest plot for comparison of postoperative WOMAC scores between the two groups.

**Figure 11:** Meta-analysis forest plot for comparison of postoperative complications between the two groups.

**Figure 12:** Meta-analysis forest plot for the comparison of the postoperative Trendelenburg sign between the two groups.

**Figure 13:** Meta-analysis forest plot for comparison of the length of limb lengthening between the two groups.

**Figure 14:** Meta-analysis forest plot for the comparison of prosthesis wear between the two groups.

**Figure 15:** Meta-analysis forest plot for the comparison of prosthesis loosening between the two groups.

**Table 1:** PubMed search strategy.

#1 Anatomic Hip Center[All Fields]
#2 High Hip Center[All Fields]
#3#1OR#2
#4 Developmental Dysplasia of the Hip[Mesh/All Fields]
#5 Hip Dislocation, Developmental OR Developmental Hip Dislocations OR
Dislocation, Developmental Hip OR Developmental Hip Dislocation OR
Developmental Hip Dysplasia OR Developmental Hip Dysplasias OR Dysplasia,
Developmental Hip OR Hip Dysplasia, Developmental [All Fields]
#6#4OR#5
#7 Arthroplasty, Replacement, Hip [Mesh/All Fields]
#8 Arthroplasties, Replacement, Hip OR Arthroplasty, Hip Replacement OR Hip
Prosthesis Implantation OR Hip Prosthesis Implantations OR Implantation, Hip
Prosthesis OR Prosthesis Implantation, Hip OR Hip Replacement Arthroplasty
OR(Replacement Arthroplasties, Hip OR Replacement Arthroplasty. Hip OR
Arthroplasties, Hip Replacement OR Hip Replacement Arthroplasties OR Hip
Replacement, Tota OR Total Hip Replacement OR Total Hip Arthroplasty OR
Arthroplasty, Total Hip OR Hip Arthroplay, Total [All Fields]
#9#7OR#8
#10#3AND#6AND#9

**Table 2:** General profile of patients included in the literature.

First author	Year	Nation	Type of study	Age (HHC/AC)	Number or hip cases (HHC/AC, years)	Gender (male/female, *n*) (HHC/AC, *n*)	Follow-up years (HHC/AC, years)	Outcome indicator
Traina [11]	2009	Italy	RS	32-76/31-67	44/44	6/30 5/32	9/9	⑦⑧⑫
Nawabi [9]	2014	America	RS	18-77	27/24	4/19 7/17	13/12	⑪⑬⑭
Ren[12]	2015	China	RS	54.4/56.2	37/35	4/25 4/24	2.2	⑤⑥⑧⑨⑬⑭
Christodoulou[8]	2010	Greece	RS	34-77.2	34/70	8/96	8.6 ± 3.5	⑤⑧⑨⑩⑪
Zhu [13]	2017	China	RS	52 ± 7/54 ± 6	33/25	4/29 3/22	2	⑤⑧⑨⑫⑬⑭
Zhang [14]	2017	China	PS	58.95 ± 11.77/57.86 ± 9.86	21/21	4/17 4/17	1	①②③④⑤⑥⑦⑧⑩⑮
Wang [15]	2018	China	RS	54.3 ± 7.6/53 ± 7.1	46/20	6/40 4/16	2	①②⑤⑥⑨⑫⑬⑭
Ge [16]	2021	China	RS	52.1 ± 5.55/54.94 ± 7.46	23/25	9/14 8/17	1.38 ± 0.24/1.45 ± 0.26	①②③④⑤⑥⑧⑨ ⑫⑬⑭
Shen [17]	2021	China	RS	50.8 ± 10.3/40.4 ± 10.2	23/19	2/21 0/19	5.8 ± 3.3/6.4 ± 3.8	⑤⑥⑧⑨⑫⑬⑭

Annotation: ① operation time; ② intraoperative blood loss; ③ postoperative drainage volume; ④ the time of going to the ground; ⑤ postoperative Harris score; ⑥ the difference in length of the lower extremities; ⑦ WOMAC scores; ⑧ postoperative complications; ⑨ postoperative Trendelenburg sign; ⑩ the length of limb lengthening; ⑪ prosthesis wear; ⑫ prosthesis loosening; ⑬ the vertical distance of the center of rotation after surgery; ⑭ the horizontal distance of the center of rotation after surgery; ⑮ hospitalization expenses. Abbreviations: HHC: high hip center technique; AC: anatomical center technique; RS: retrospective study; PS: prospective case series.

The article "Meta-analysis of the Efficacy of the Anatomical Center and High Hip Center Techniques in the Treatment of Adult Developmental Dysplasia of the Hip" was published in 2022. Journal: Biomed Res Int.

**Table 3:** The included retrospective studies were assessed for quality using the Newcastle–Ottawa scale.

First author/year	Selection of population (fraction)	Comparability between groups (fraction)	Outcome measure (fraction)	Overall score (fraction)	Quality rating
Traina, 2009 [11]	4	0	1	5	Middle
Nawabi, 2014 [9]	4	0	1	5	Middle
Christodoulou, 2010 [8]	3	0	2	5	Middle
Ren, 2015 [12]	4	0	1	5	Middle
Zhu, 2017 [13]	3	2	1	6	Middle
Wang, 2018 [15]	3	2	1	6	Middle
Ge, 2021 [16]	3	2	2	7	Highness
Shen, 2021 [17]	3	2	1	6	Middle

Annotation: the full score of the Newcastle–Ottawa scale was 9 points; ≥7 was considered high-quality literature; 5-6 points was divided into medium-quality literature; <5 points was considered low-quality literature.

## Data Availability

All data used to support the findings of this study are included within the article.
